RETRACTED

# Comparative value of clinical, cytological, and histopathological features in feline mammary gland tumors; an experimental model for the study of human breast cancer

**DOI:** 10.1186/1746-1596-8-136

**Published:** 2013-08-13

**Authors:** Radmehr Shafiee, Javad Javanbakht, Nahid Atyabi, Alimohammad Bahrami, Danial Kheradmand, Reyhaneh Safaei, Farshid Khadivar, Ehsan Hosseini

**Affiliations:** 1 Graduate, Faculty of Veterinary Medicine, Tehran University, Tehran, Iran; 2 Department of Pathology, Faculty of Veterinary Medicine, Tehran University, Tehran, Iran; 3 Paraveterinary Faculty of Ilam, University of Ilam, Ilam, Iran; 4 Graduate Student of Islamic Azad University of Mashhad, Faculty of Medicine, Mashhad, Iran

**Keywords:** Pathology, Cytology, Cats, Mammary gland, Tumours

## Abstract

**Background:**

The diagnosis of breast lesions is usually confirmed by fine-needle aspiration cytology (FNAC) or histological biopsy. Although there is increasing literature regarding the advantages and limitations of both modalities, there is no literature regarding the accuracy of these modalities for diagnosing breast lesions in high-risk patients, who usually have lesions detected by screening. Moreover, few studies have been published regarding the cytopathology of mammary tumors in cats despite widespread use of the animal model for breast cancer formation and inhibition. The objective of the present study was to evaluate the diagnostic interest of cytological and histopathological analysis in feline mammary tumours (FMTs), in order to evaluate its possible value as an animal model.

**Methods:**

The study was performed in 3 female cats submitted to surgical resections of mammary tumours. The mammary tumours were excised by simple mastectomy or regional mastectomy, with or without the superficial inguinal lymph nodes. Female cats were of different breeds (1 siamese and 2 persians). Before surgical excision of the tumour, FNA cytology was performed using a 0.4 mm diameter needle attached to a 8 ml syringe held in a standard metal syringe holder. The cytological sample was smeared onto a glass slide and either air-dried for May-Grünwald-stain and masses were surgically removed, the tumours were grossly examined and tissue samples were fixed in 10%-buffered-formalin and embedded in paraffin. Sections 4 μm thick were obtained from each sample and H&E stained.

**Results:**

Cytologically, atypical epithelial cells coupled to giant nucleus, chromatin anomalies, mitotic figures, spindle shape cells, anisocytosis with anisokaryosis and hyperchromasia were found. Histologically, these tumors are characterized by pleomorphic and polygonal cell population together with mitotic figures, necrotic foci and various numbers inflammatory foci. Also, spindle shaped cells, haemorrhage localized in the different regions, local invasiveness and enlarged nuclei were observed. The samples included 3 tumors of mammary glands mammary tumors were complex carcinomas (n = 2) and adenocarcinoma (n = 1). The histological grades of the 3 cases were as follows: grade II, (1/3); grade III, (2/3) with high mitotic index. The preferential localization of mammary neoplasms was in the inguinal lobe (1/3 case) and abdominal lobes (2/3 cases). Furthermore, 1case of the inguinal mass affected the left caudo-inguinal lobe and 2cases right cranio and caudo abdominal lobes.

RETRACTED

**Conclusion:**

The study concluded that cytology could be used as a quick, rapid, field diagnostic technique in combination with histopathology for the diagnosis of feline mammary tumors (FMTs). Our findings in feline MTs indicate that FMTs could be useful as an animal model of human breast cancer. Moreover, because of the similarity of the cytohistopathological findings in the human and feline mammary gland tumours, it is possible to use the same cytopathological criteria applied in human pathology for the diagnosis of feline mammary gland tumours.

**Virtual slide:**

The virtual slide(s) for this article can be found here: http://www.diagnosticpathology.diagnomx.eu/vs/2047361423103295

## Background

Breast cancer is the most frequent occurring tumor in humans. Mammary tumours (MTs) are among the most common neoplasms in both cats and dogs, but the prevalence of malignant histological types is far higher in cats (ratio of malignant: benign is at least 4:1). Feline MTs comprise approximately 11% of feline non-integumentary neoplasms, are more commonly malignant than benign, and carry a poor prognosis attributable to a high probability of local recurrence and metastasis [1,2].

Feline mammary complex carcinoma and adenocarcinoma are one of the most common feline neoplasms and represent an important cause of mortality. The incidence and the morbidity of these tumors have been demonstrated to be very high because their biologic behavior is characterized by rapid growth, high proliferation rates, and capability to metastasize to regional lymph nodes and distant organs [3-5].

MTs are commonly observed in female cats [6]. Between 80% and 96% of these tumors are malignant and very aggressive [7,8], MTs are an important cause of mortality, especially in middle-aged and elderly females. The interval between feline mammary carcinoma detection and death varies from <6 to 12 months [8]. Several factors, including age, diameter of the primary lesion, the presence of histologically tumor-positive lymph nodes, mitotic count, extent of necrosis, and complete surgical excision, are independently correlated with post-surgery survival time.

RETRACTED

A number of new methods are therefore tested within tumor pathology to improve the diagnostic and prognostic accuracy. To make a diagnosis, a number of clinical and paraclinical tests are used because it is essential to find the most aggressive malignant tumors that need radical surgery and supplementary treatment as soon as possible. After excision, a hematoxylin-eosin stain is often used to provide a histopathological diagnosis, but even though this is performed by experienced pathologists, the disorderly structure of some mammary tumors may cause confusion and may lead to an erroneous diagnosis of malignancy [9-12].

Fine needle aspiration cytology (FNAC) is a method largely used to obtain samples for cytological diagnosis in several organs. When applied to mammary gland lesions, the method shows good diagnostic accuracy. Moreover, it is a simple, rapid and low cost method, with minimal risk for the patien [11,12]. In veterinary medicine, the use of cytology as a diagnostic method is very recent and has been growing in the last 20 years [13].

Despite this copious literature, there have been few reports of mammary tumors in feline. Retrospective reports have described the epidemiologic characteristics, gross morphology, and microscopic features of both benign and malignant mammary tumors [14].

To the best of our knowledge, the literature lacks information on the cytohistopathological profile of mammary tumors in this species. The present study was designed to morphologically and cytopathologcally describe spontaneous mammary gland tumors in cat. We also considered the usefulness of tumor grading as a prognostic indicator.

## Methods

### Characterization and clinical features of cases

Three cats were undergone surgery at the Department of Veterinary Clinic, School of Veterinary Medicine, University of Tehran, from July 2012 to April 2013 were initially included in the study. The animals, aged 6, 10 and 16 years, showed with or without clinical or radiological evidence of distant metastasis. Female cats were of different breeds (1 Siamese, and 2 Persian).

All subjects received a total mastectomy, and surgical excision specimens were fixed for 48 hours in buffered formalin, routinely processed, and examined histologically. Sections were routinely stained with hematoxylin and eosin, and lesions were classified accordingly to the World Health Organization Histological Classification of the mammary tumours of the Cat [15].

### Cytohistological and surgical evaluation

Before surgical excision of the tumour, FNAC cytology was performed using a 0.4 mm diameter needle attached to an 8 ml syringe held in a standard metal syringe holder. The cytological sample was smeared onto a glass slide and either air-dried for May-Grünwald-stain. Subsequently, cats were induced with propofol (2 mg/kg, IV, Propofol, Abbott) and anaesthetized with isoflurane (2-3%, Isoflurane, Adeka) and masses were surgically removed, the tumours were grossly examined and tissue samples were fixed in 10%-buffered-formalin and embedded in paraffin. Sections 4 μm thick were obtained from each sample and H&E stained. The cytopathological criteria adopted were those proposed by Bibbo (1997) [16].

RETRACTED

### Classification of tumors

Mammary neoplasms were classified by size according to the World Health Organization Clinical Staging System TNM [17], as T_1_ (<3 cm maximum diameter), T_2_ (3–5 cm maximum diameter) and T_3_ (>5 cm maximum diameter). In cases of multiple tumours, the largest one was used as the basis for classification.

Representative portions of each tumor were fixed in 10% neutral buffered formalin and were routinely embedded in paraffin. Four-micrometer-thick sections were stained with hematoxylin and eosin (HE) for histologic evaluation.

### Grading of tumors

Histologic tumor grading was performed on HE-stained sections using a previously described classification [18], the grade for each case was derived from an assessment of (1) tubule formation, (2) nuclear pleomorphism, and (3) mitotic counts, each feature being scored 1 to 3 points. The scores were then added to obtain the tumour grade, as follows: 3–5 points, well-differentiated (grade I); 6–7 points, moderately differentiated (grade II); 8–9 points, poorly differentiated (grade III). Grading was carried out by a veterinary pathologist and without prior knowledge of the results, and confirmed by a second pathologist.

## Results

### Macroscopic findings and tumour size

The macroscopic specifications of the multifarious mammary masses were summarized in the Table 1. The preferential localization of mammary neoplasms was in inguinal lobe (2 cases) and abdominal lobes. Furthermore, 1 case of the inguinal mass affected the caudo-inguinal lobe and % 67 cranio and caudo abdominal lobes. Eventually, 2 cases of tumour masses were found in the right mammary lobes and 1 case in the left mammary lobe.

**Table 1:** Macroscopic characteristics of the mammary masses in the 3 females’ cats

**Case n°**	**Breed**	**Age**	**Tumour localisation**	**Weight (g)**	**Size (cm)**	**Consistency**
1	Persian	6	Left caudo- inguinal lobe	13	2x2x1.8	Hard
2	Siamese	10	Right caudo- abdominal lobe	28	4x3x2.6	Hard
3	Persian	16	Right craino-abdominal lobe	150	11x10x9	Hard

According to their maximum diameter, the tumours were classified as T_1_ in 1/3 (<2 cm maximum diameter), T_2_ in 1/3 (<4 cm maximum diameter) and T_3_ in 1/3 (<11 cm maximum diameter) cats.

RETRACTED

### Cytology evaluation

All the tumor masses were divided into two cytologic groups: adenocarcinoma (2/3 cases) and carcinoma (1/3 cases). Cytologically, some nuclear anomalies were identified such as double nucleus in 2 samples of malignant tumours (Figure 1A), giant nucleus in 2 samples, mitotic figures in 3 samples and abnormal chromatin structures in 3 samples (Figure 2D). In 1 case spindle shaped cells was associated with tumour cells (Figure 2B, C and D). Furthermore, clusters of cells with anisocytosis,anisokaryosis and hyperchromasia were observed (Table 2 and Figure 2A).

**Figure 1:** **Evaluation of accuracy of fine needle aspiration cytology and histopathology for diagnosis of feline mammary tumours. A**: Malignant multinucleated mammary epithelial cell; nuclei exhibit nuclear criteria of malignancy; nuclei super imposed and in different focal planes. May-Grunwald-Giemsa staining method, 1000X. **B**: Cells exhibit variable numbers of mitoses are found; or the second populationof cells may have oval to fusiform vesicular nuclei with an extensive amount of eosinophilic cytoplasm and distinc cell margins (H&E, X 400). **C**: Solid adenocarcinoma; The presence of neoplastic, mitotic and inflammatory cells (H&B, X 200.), **D**: Hemorrhage foci and the central necrotic areas are interpreted as an indication that the neoplastic cells are growing faster and that there is therefore a higher risk of progressionto invasive carcinoma (H&E, X100).

**Figure 2:** **Evaluation of accuracy of fine needle aspiration cytology for diagnosis of feline mammary tumours. A:** Malignant epithelial cells; nuclei exhibit nuclear criteria of malignancy (variable size, macronucleoli); nuclei superimposed and in different focal planes, together with variation in cell (*anisocytosis*) and nuclear. (*anisocytosis*) size are present and abundant vacuoles, May-Graun-Giemsa staining method, 1000X. **B**: Cytological appearance of spindle shape cells (tomour from the cat n°1) and pleomorphic malign epithelial cells in adenocarcinoma, *May*-*Grünwald Giemsa* (MGG) staining method, 1000X. **C** and **D**: Myoepithelial cells (spindle shape) with abundant chromatin granules, irregular in shape, and unevenly dispersed throughout nucleus in adenocarcinoma, May-Grunwald-Giemsa, X 400 and X 1000.

**Table 2:** Cytological analysis of pre-operative fine needle aspirates from the mammary neoplasms of the 3 females cats

**Case n°**	**Giant nucleus**	**Spindle shaped cells**	**Abnormal chromatin**	**Mitotic rate**	**Double nucleus**	**Anisocytosis**	**Anisokaryosis**	**Hyperchromasia**
1	+	+	+	+	+	+	+	+
2	^_^	^_^	+	+	^_^	+	+	+
3	+	^_^	+	+	+	+	+	+

RETRACTED

### Histopathological characteristics of the tumours

The histological grades of the 3 cases were as follows: grade II, 1/3 case; grade III, 2/3 cases with high mitotic index. The relationship between tumour grading and histological type is presented in Table 1. Of the 3 cats in which mammary examination was performed, 1 had moderately differentiated grade II (1 complex carcinoma) and 2 had poorly differentiated grade III (1 solid adenocarcinoma and 1 complex carcinoma) (Table 3).

**Table 3:** Cytological and histopathological analysis of pre-operative and sampled during surgery from the mammary neoplasms of the 3 females felines together with signalment of cats

**Case n°**	**Grade type**	**Cytological type**	**Cytological classification**	**Histopathological type**	**Histopathological classification**
1	III	Carcinoma	Malignant	Complex carcinoma	Malignant
2	II	Adenocarcinoma	Malignant	Complex carcinoma	Malignant
3	III	Adenocarcinoma	Malignant	Solid adenocarcinoma	Malignant

The samples under evaluation included 3 tumors of mammary glands. Results showed that all samples were malignant 100% (n = 3) of mammary tumors were carcinomas and adenocarcinoma respectively.

All the tumor samples were divided into two histopathologic groups: solid adenocarcinoma (1 case) (Figure 1C) and complex carcinoma (2 cases).

Of the 3 FMTs included, all cases exhibited a range of morphologies, a highly pleomorphic cell population and polygonal were a prominent feature of all neoplasms. Furthermore, 1of the 3 case was composed of highly cellular areas with a homogeneous population of spindle cells. Moreover, a high mitotic rate was identified in 3 cases, with atypical mitoses conspicuous in all tumours (Figure 1B). In addition, 2 of the 3 FMTs cases showed necrotic foci (Figure 1D) and infiltrates of various numbers inflammatory foci primarily consisting of lymphocytes, plasma cells, and neutrophils cells. Also, all cases exhibited haemorrhage localized in the different regions of the tumor tissue (Figure 1D). According to local invasiveness, 67% of the tumours (2 out of 3) were observed (Table 4).

**Table 4:** Histopathological analysis of mammary tumours sampled during surgery in the 3 females cats

**Case n°**	**Pleomorphic and polygonal cell population**	**Spindle shaped cells**	**Mitotic figures**	**Necrotic foci**	**Various numbers inflammatory foci**	**Haemorrhage localized in the different regions**	**Local and vascular invasion**	**Enlarged nuclei**
1	+	+	+	+	^_^	+	^_^	+
2	+	^_^	+	+	+	+	+	^_^
3	+	^_^	+	^_^	+	+	+	^_^

RETRACTED

## Discussion

All the cases reported in this study have similar morphologic features to cases observed in women's breast tumors [19-23]. Mammary neoplasias are the third most frequent neoplasias in cats, accounting for 12% of all feline tumors [24,25].

Fine needle aspiration cytology of the breast has a high range of accuracy (72–99%) [8,10], in the diagnosis of malignancy and its sub typing. Despite this, some rare lesions create problems at cytodiagnosis. Accuracy of cytodiagnosis of malignant breast tumors is very important to know the exact line of treatment preoperatively. Histologically, 25–30% of epithelial malignancies are in the group of specialized breast carcinoma like lobular, papillary, apocrine, tubular, cribriform, medullary, mixed, etc. [10,11]. In order to deciding the best type of treatment, sub typing of breast tumors using aspiration cytology is useful. If tumors are of low malignant potential, options for conservative breast carcinoma treatment are being available for the patient [9,10]. However, it is not always possible to label the exact subtype on aspiration cytology without correlating the clinical and histopathological findings. We performed a validity study to further characterization of sensitivity and specificity values as well as the accuracy of FNA cytology in the diagnosis of feline MTs.

In some studies, the fine needle aspiration cytology specimens contained many individual bizarre, multi-nucleated, and/or giant cells having hyperchromatic pleomorphic nuclei, prominent nucleoli, and relatively abundant cytoplasm, admixed with numerous mitotic figures in a hemorrhagic or inflammatory background in human. A small amount of sheet-like or three-dimensional clusters of malignant cells coexisted [26-30].

In our study, we found 100% cytological and histological diagnostic agreement. These results are similar when compared with results of studies of human breast lesions published by Choi et al. [31] and Ciatto et al. [32]. They described high levels of agreement between cytological and histological diagnoses, ranging from 64.8% to 74.1%. In addition, when the authors excluded the inconclusive cases, their level of agreement increased to 93.1 and 96.7%, respectively. The results were at variance with findings of Bofin et al. [11], who reported 84.6% of correlation between cytological and histological diagnoses of mammary tumours.

Histopathologic examination was considered as the gold standard for the diagnosis of feline MTs. The histological analysis of feline MTs usually includes a spindle cell component Haziroglu et al., 2010, present spindle shaped cells reported in one case of malignant mixed tumour and in one case of complex carcinoma [33]. In the present study, spindle shaped cells were encountered in one case of complex carcinoma in accordance with previous reports.

RETRACTED

Histologically, carcinomas differed from benign mammary tumors in at least one of the following features: atipia in the epithelial component of the tumor growth, infiltrative growth, high mitotic activity and cellularity, and/or necrosis. In general, the malignant mammary gland tumors were mostly well or moderately differentiated. In current study, features of anaplasia such as bizarre mitotic figures, an increased nuclear/cytoplasmic ratio, and hyperchromatic nuclei were observed in our feline MACs.

Our histological findings resembled those included in the World Health Organization’s classification of mammary tumors of the dog and cat [15]. Other authors have used this classification system to classify mammary tumors in other species [34,35]. In effect, we believe that pathologists and clinicians should routinely use this system to standardize, interpret, and accurately reproduce research results. In our study, all tumors were malignant, 2 were complex carcinoma (case Nos. 1 and 2), and also, 1 case was a adenocarcinoma (case No. 3).

Neoplastic, multinucleated giant cells are common cell type in feline carcinomas and adenocarcinoma and are associated with tumors of a high histologic grade [36]. Considering these results in present study, neoplastic, multinucleated giant cells may be an important source of malignant factor that could increase the growth of carcinomas. These results, together with the pleomorphic cellular appearance, indicate a poorly differentiated tumor, in accordance with previous reports [37].

A histologic grading system, based on assessing the degree of tubule formation, mitotic activity, and nuclear pleomorphism, has been used for canine and feline mammary carcinoma [23]. The histologic grade of malignancy is determined by the sum of individual scores for these features and is of prognostic significance. Through the use of this system, the masses in the current study were categorized as moderately and poorly grade. The low-grade malignancy and the lack of evidence of infiltration correlate well with the slow clinical progression in these cats.

This study supports the previously reported lack of correlation between survival period of cats with their age, breed, sex, or type of surgical excision of the tumor [38,39]. The age of affected cats, gross appearance of the tumors, as well as prevalence of benign versus malignant mammary tumors in this study were similar to those in previous reports [4,7,38-44]. The present study supports the previously reported higher prevalence of adenocarcinoma in abdominal mammarylobe [33,44,45]. However, some authors have reported that abdominal lobe [43,45,46] are more commonly affected by tumors, whereas others have found inguinal lobes to be involved more often [4].

RETRACTED

In summary, this study described some clinical-cytopathologic features of 3 cats with histologic features that correspond to feline MACs of the mammary gland in women. To the best of our knowledge, this is the first report describing the clinico-cytohistopathologic features of these tumors type in Siamese and Persian feline mammary glands in Iran.

## Conclusions

All cases of feline MACs of the mammary gland herein reported were associated with clinical-cytopathologic features of high biologic aggressiveness and low survival rate and should be classified as an independent histologic type of FMAC. These results also suggest that FMAC, on the basis of histologic and clinical outcome, it is a good animal model to study women's breast cancer.

### Ethical approval

All experimental protocols were approved by the local animal care committee in accordance with undergone surgery at the Department of Veterinary Clinic, School of Veterinary Medicine, University of Tehran, from July 2012 to April 2013 were initially included in the study and office regulations. All experiments and animal housing adhered to the Guideline for Care and Use of Laboratory Animals of the Institute of Clinic Animal Resources, National Research Council (2012). Experimental procedures were approved by the ethical review board for animal experiments at the University of Tehran (approval number; S-2010 MED-29). The animals, aged 6, 10 and 16 years, showed with or without clinical or radiological evidence of distant metastasis. Female cats were of different breeds (1 Siamese, and 2 Persian).

## Abbreviations

FNA: Fine needle aspiration; FMTs: Feline mammary tumours; MTs: Mammary tumours; TNM: Classification of malignant tumours; HE: Hematoxylin and eosin; MACs: Mammary carcinomas and adenocarcinoma. 

## Competing interests

The authors declare that they have no competing interests.

## Authors’ contributions

NA and RSH participated in the histopathological evaluation, performed the literature review, acquired photomicrographs and drafted the manuscript and gave the final histopathological diagnosis and designed and carried out all the experiments. JJ is the principal investigator of the laboratory in which the research was performed and contributed to the interpretation of the data and writing of the manuscript. AMB, DKH,RS,FKH and EH edited the manuscript and made required changes and wrote the manuscript. All authors have read and approved the final manuscript.
